# Development and Optimization of a New Chemoenzymatic Approach for the Synthesis of Peracetylated Lactosamine (Intermediate for the Synthesis of Pharmacologically Active Compounds) Monitored by RP- HPLC Method

**DOI:** 10.15171/apb.2017.037

**Published:** 2017-06-30

**Authors:** Qais Ibrahim Abualassal, Khaldun Mohammad Al Azzam, Zead Helmi Abudayeh, Loay Khaled Hassouneh

**Affiliations:** ^1^Faculty of Pharmacy, Isra University, Amman, Jordan.; ^2^Department of Drug Sciences, University of Pavia, Italy.; ^3^Preparatory Year Department, Al-Ghad International Colleges for Applied Medical Sciences, 11451 Riyadh, Kingdom of Saudi Arabia.

**Keywords:** Glycosylation reaction, Chemo-enzymatic synthesis, Regioselectivity, High performance liquid chromatography, Flash column chromatography, Candida rugosa

## Abstract

***Purpose:*** To describe a chemoenzymatic approach joining an enzymatic regioselective hydrolysis of peracetylated N-acetyl-α-D-glucosamine (**A**) with a mild controlled acyl relocation which resulted 2-acetamido-2 deoxy-1,3,6-tri-O-acetyl-α-D-glucopyranose (**1B**).

***Methods:*** Immobilization of lipase on decaoctyl (DSEOD) and octyl-agarose (OSCL) was carried out as reported by the work of Bastida et al. The newly developed RP-HPLC method for examining the enzymatic hydrolysis was carried out isocratically utilizing a HPLC system.

***Results:*** The new approach resulted the target compound (**B**) in 95% yield after purification utilizing flash column chromatography. Candida rugosa-lipase immobilized ondecaoctyl-sepabeads was the best catalyst in terms of activity and region-selectivity in the hydrolysis of substrate (**A**), delivering the deacetylation at C6 position (98% general yield). Also, a reversed-phase high-performance liquid-chromatographic (RP-HPLC) method for controlling the region-selective hydrolysis of peracetylated N-acetyl-α-D-glucosamine (**A**) with a mild monitored acyl movement which led to 2-acetamido-2-deoxy-1,3,6-tri-O-acetyl-α-D-glucopyranose (**1B**) has additionally been developed. The developed RP-HPLC method was utilized as fingerprints to follow the hydrolysis of substrate (A) and to determine its purity and additionally yield. Furthermore, the acquired compound (**B**) was further purified by flash chromatography. Compound (**B**) was further characterized utilizing ^1^HNMR and mass spectrometry.

***Conclusion:*** An efficient chemoenzymatic procedure to optimize the preparation of peracetylated lactosamine B containing acetyl ester as extraordinary protecting group is presented. Compound **B** is a significant intermediate for the synthesis of pharmacologically active compound (e.g. complex oligosaccharides for biochemical, biophysical, or biological examinations). Besides, reaction monitoring utilizing HPLC proposes more exact information than spectroscopic methods.

## Introduction

Carbohydrates are viewed as a key part in various biological processes. Given their differing difficulty in all cells, it is not surprising that glycans have various assorted part in different physiological processes. The physiological processes are made out of sophisticated multi-cell living organism form. Honestly, a generous number of bioactive compounds are glycosylated and the sugar moiety is considered as a key for their bioactivity.^1^ Of them, glycoproteins found in cell–cell recognition of various pathologies are of remarkable interest.^2^ Actually, oligosaccharides found in glycoproteins are recognized by lectin receptors, the key part for carbohydrate-mediated recognition actions.^3^ For example, lacto oligosaccharides series are incorporated into a couple of structures with high biological concern (e.g., glycolipids and glycoproteins) (Figure 1).^4-6^

The destiny of carbohydrate science will be great by the use of its products. The access to oligosaccharides by separation from natural sources is believed tedious and subsequently it gives simply little material that consistently needs the targeted level of purity. The synthesis of high purity oligosaccharides is considered a challenge. Additionally, it is critical for improvement of glycobiology branch.^7^ The absence of fruitful and successful methods for synthesis decreased the usage and the examination of oligosaccharides for therapeutic and diagnostic applications. The preparation of monodeprotected sugar is one of the basic building stones in accomplishing complex oligosaccharides.^8,9^

Due to the complexity of structure as well as variability of oligosaccharides, it has been highlighted more than in case of proteins or DNA. Moreover, they are not controlled by genes and complex polymer, thus they are not valid techniques. For example, PCR for the nucleic acids or recombinant DNA procedure for proteins, found in bacteria, is profitable for the manufacturing on a quantitative scale.^10^ Therefore; the preparation of large amounts of carbohydrates starting from natural sources is suitable to conduct studies or even utilize them as pharmacological substances. Additionally, the advances in glycobiology are constrained because of the absence of efficient techniques to characterize and sequence polysaccharides.^7^

**Figure 1:** Oligosaccharides as a key component for carbohydrate determinates highly expressed on the surface of malignant cells.

The advances in chemical synthesis of carbohydrates to find more successful, effective and automated techniques is crucial for the development in glycobiology. It is vital to be used in oligosaccharides in therapeutic and diagnostic area. Herein, it should be highlighted that the synthesis of large amounts of oligosaccharides can improve the production of medication more effectively than the relating natural products.^11-13^

The online/inline evaluation is viewed as a capable tool for controlling and monitoring organic reactions through scale-up step. In addition, the kinetic data obtained from these reviews not just permits control of reactions in routine production but also encourages the design of robust methods and subsequently better idea of the reaction mechanisms.^14^ Also, it decreases the tedious work prior reaction controlling through expelling the requirement for manual sampling. This methodology is valuable in conditions where a percentage rate of the reaction compositions are labile or even where the reaction mixture may be dangerous to operator.^15,16^

Flash chromatography technique offers a quick and efficient strategy for separation of mixtures requiring rational resolution.^17^ Furthermore, it can be applied for both modes namely; normal phase and reversed phase sepration.^18^ Other advantages such as high flow rate with low pressure, thus good separation in a short time and under a reasonable chromatographic conditions could be achieved.^17^

Since long time, our potential research group has been focusing on the mono-protective approach which is necessary for the synthesis of oligosaccharides.^19^ In this work, we investigated, optimized and developed another chemoenzymatic approach for the synthesis of oligosaccharides. The last is considered a key intermediate in the regioselective enzymatic hydrolysis of peracetylated pyranoses that catalyzed by the immobilized lipases. Literature review reveals that no reports have been reported for the chemoenzymatic approach for the synthesis or optimization of peracetylated lactosamine (PL) or even using reversed-phase high performance liquid chromatography (RP-HPLC) and flash chromatography methods as monitoring tools for the hydrolysis and purifying, respectively.

In the present work, we concentrated on the development and optimization of another chemoenzymatic approach for the synthesis of PL. In addition, the subsequent acyl movement of the hydrolyzed product to obtain the particularly monodeprotected acyl-pyranose holding a free hydroxyl group at C4 position has additionally been examined. These synthons were successfully and effectively used as an important part in the synthesis of oligosaccharides. The immobilized acetyl xylan esterase (ACEXE) has also been used as another approach for the hydrolysis of substrate **A**. Also, sensitive and direct method is considered important to screen the hydrolysis of substrate **A** and to purify the obtained product **B**. Along these, RP-HPLC and flash chromatographic methods have also been developed in this work.

## Materials and Methods

### Reagents and chemicals

The octyl-sepharose CL-4B (OSCL) and decaoctyl Sepabeads ECOD/S (DSEOD) were purchased from Amersham Pharmacia Biotech Co. (Uppsala, Sweden). *N*-acetyl-D-glucosamine (C_8_H_15_NO_6_), β-D-galactose pentaacetate (C_16_H_22_O_11_), lipase from *Candida rugosa lipase* (CRGL), HPLC grade acetnitrile (CH_3_CN) and methanol (CH_3_OH), ethyl acetate CDCl_3_-d, sulfuric acid (H_2_SO_4_), dichloromethane (CH_2_Cl_2_), ethanol (CH_3_CH_2_OH), anhydrous sodium sulfate (Na_2_SO_4_), tetramethylsilane (TMS) (Si(CH_3_)_4_), triethylamine ((C_2_H_5_)_3_N), sodium chloride (NaCl), boron trifluoride diethyl etherate (BF_3_·O(C_2_H_5_)_2_), sodium azide (NaN_3_), toluene (C_6_H_5_CH_3_), and sodium hydroxide (NaOH), were obtained from Sigma-Aldrich (Milan, Italy). Immobilized acetylxylan esterase (ACEXE) (*Bacillus pumilus*) was a kind gift from ACS Dobfar SPA. All other reagents were of high analytical grade. Substrates that were not commercially available were synthesized in our lab utilizing reported protocols.

### Immobilization of CRGL on DSEOD and OSCL

Immobilization of lipase on DSEOD and OSCL was done based on the protocol described by Bastida *et al*.^20^ In brief, an exact amount of enzymatic extract was diluted with the aid of phosphate buffer solution (25 mM, pH 7) and then kept under continuous mixing for 30 min. An exact amount of DSEOD and OSCL, (conditioned previously with the same buffer solution and then dried on glass funnel for 1 min) was added to the enzymatic solution in a ratio of (1:10, v/v). After that, the suspension was kept under gentle mixing at room temperature for 3 h. The route of immobilization was tested through Bradford assay method.

Once finished, the enzymatic preparation was isolated using filter paper on glass funnel, washed out using distilled water and with a solution of sodium azide of concentration 0.02% w/v. The yield was assessed through the determination of the weight in mg of protein found in the supernatant. The activity of the enzymatic solution was assessed using ethyl-butyrate test (section 2.3).

### Estimation of lipase activity using ethyl butyrate assay test

A 16 mL solution of phosphate buffer of concentration100 mM, pH 7 was mixed with 4 mL of ethyl butyrate. Then, 100 μL of free enzyme or 50 mg of the enzymatic solution was poured to the solution prepared under vigorous mixing. Throughout the assay (15-20 min), the pH was controlled and kept constant during the addition of NaOH solution (50 or 100 mM) with the aid of programmed titration pH-meter (Metrohm 718 STAT Titrino, Herisau, Switzerland). In light of the consumed amount of NaOH solution, the activity was estimated and expressed in U/g or U/mL.

### Procedure for enzymatic hydrolysis in aqueous medium

The enzymatic hydrolysis of **A** was achieved in 50 mM phosphate buffer and with the aid of 20% acetonitrile (pH 4, and 5) to assure full solubilization through mechanical blending. The reaction began at ambient temperature after addition of the immobilized enzyme solution. The pH was kept constant, during the reaction, via programmed titration. The reason of keeping pH constant is to avoid the chemical acyl movement that may happen in the per-*O*-acetylated carbohydrates hydrolysis.^21^

The course of the hydrolysis was controlled by HPLC. The products were evaluated using the synthetic standards isolated. After the whole usage of the substrate, the reaction was stopped utilizing biocatalyst and the generated products were isolated by extraction with the aid of ethyl acetate. The organic layer was dried over anhydrous sodium sulfate, then filtered, and dried under vacuum. The residue was further purified by flash chromatography, and after that it has been subjected to NMR spectroscopy and mass spectrometry for characterization.

### Chemical acyl migration/movement 

The immobilized biocatalyst was separated by normal filtration. The solution that contains 6-OH derivative **1A** was incubated at pH 9 and 4°C to facilitate the acyl migration from position C4 to C6. RP-HPLC was used, as mentoring tool, to control obtaining the targeted substrate **1B**. At that point, the solution was saturated utilizing sodium chloride and subsequently separated by ethyl acetate. Anhydrous sodium sulfate was used as drying agent to dry the organic layer, then separated and afterward dried under vacuum. The crude products (unrefined) was purified utilizing flash chromatography.

### Synthesis of 1A

Enzymatic hydrolysis method was followed for the synthesis of this compound as prescribed by the earlier protocol. Moreover, silica gel flash chromatography was applied for purification of the crude product. A mixture of methanol/dichloromethane using the following ration 5:95,v/v was used for successful elution. The obtained yield (98%) was determined after purification by flash chromatography. Retention factor (R_f_) was 0.32. HPLC chromatographic conditions applied were 20% acetonitrile in phosphate buffer, 10 mM, pH 4, and at flow rate of 1.0 mL/min. Retention time (t_R_) was 5.70 min.

### Synthesis of 1B

The method of acyl migration/movement mentioned above was adopted for the synthesis of this compound. Moreover, silica gel flash chromatography was applied for the purification of the crude product using a mixture of methanol/dichloromethane (5:95, v/v) to provide the desired glassy white solid product. The yield obtained was 90% after purification by flash chromatography. HPLC chromatographic conditions applied were 15% acetonitrile in phosphate buffer, 10 mM, pH 4, and at flow rate of 1.0 mL/min. t_R_ was 7.50 min.

### Synthesis of product B

A 1.77 g or 3.597 mmol of 2,3,4,6-tetra-O-acetyl-α-D-galactopyranosyltrichloro acetimidate (2) and 0.5 g or 1.44 mmol of **1B** were dissolved in 10 mL CH_2_Cl_2_. After that, boron trifluoride diethyletherate (0.346 mL or 2.769 mmol) was added in the presence of activated molecular sieves (4Å). Then, mixing at room temperature and under nitrogen was done. After mixing for 5 h, the reaction was quenched by adding 0.39 mL of triethylamine. After that the residue was further purified utilizing flash column chromatography using a mixture of methanol/toluene/ethyl acetate, 1:6:8, v/v to give the requested product. The yield was 95% and R_f_ 0.24.

### Biocatalysts recycling

To look at the reusability or reusing of the immobilized enzymes specified before, the hydrolysis of **A** was examined under comparable conditions. As the highest conversion was accomplished, the reaction mixture was filtered under reduced pressure, washed and after that the immobilized biocatalyst was reused for the following reaction.

### ^1^H NMR and mass spectrometry

The ^1^H NMR spectra were conducted in deuterated chloroform (CDCl_3_) for **B**. The analysis was achieved at 298 K, 400.1 and 100.6 MHz using a Bruker Avance 400 MHz Spectrometer (Bruker, Karlsruhe, Germany). The Bruker Avance instrument was equipped with a 5 mm BBI inverse gradient probe. Also, the spectrometer used was equipped with a Topspin Programming Package on a workstation running Windows Operating System. Chemical shifts were recorded based on the internal reference TMS. The purified **B** was dissolved in CDCl_3_. The products obtained by enzymatic hydrolysis were characterized by 2D-Cozy (Correlated Spectroscopy), HSQC (Heteronuclear Single Quantum Correlation) and HMBC (Heteronuclear Multiple Bond Correlation). In addition, 2D NMR was carried out to allocate the correct position of the hydrolysis.

### TLC

TLC was carried out on a 0.2 mm layer silica gel pre-coated aluminum sheets purchased from Merck, Darmstadt, Germany. The mobile phases used in TLC analysis comprise of methanol/ethyl acetate/toluene of ratio 16:8, v/v/v and methanol/dichloromethane of ratio 5:95, v/v were utilized to track the preparation of **1B** and **B**, respectively. The spots on TLC were identified by spraying the plates with a mixture consisting of 5% H_2_SO_4_ solution in ethanol, then by warming to 150 ^°^C. Silica gel 60 of 40–63 μm, was purchased from Merck and utilized for flash chromatography. R_f_ values were 0.24 and 0.30 for the **1B** and **B**, respectively.

### RP-HPLC for monitoring the enzymatic hydrolysis

A new RP-HPLC method was applied for controlling/monitoring the enzymatic hydrolysis process. It was carried out using isocratic elution. The HPLC system (model L-7100) used (Merck-Hitachi, Darmstad, Germany) equipped with a pump (model, L-7100), an interface (model, L-7000), a diode array detector (model, L-7400), an auto sampler (model, L-7200) with a 20 μL sample loop, a degasser (model, L-7612) and a high pressure gradient mixer. LaChrom Software (version 3.2.1) was used to record the data analysis. Separation was achieved utilizing a Phenomenex C-18 column (250 x 4.6 mm, i.d., 5 μm) (Chemtek Analitica, Anzola Emilia, Italy). Other chromatographic conditions such as column oven at 25°C and at a detection wavelength of 220 nm were applied. The flow rate was 1.0 mL/min using a mixture of 20 and 15% acetonitrile in 10 mM phosphate buffer, adjusted to pH 4 as a mobile phase for **1A** and **1B**, respectively. t_R_ were 5.70, and 7.50 min for **1A** and **1B**, respectively (chromatograms are not shown).

### Flash chromatography 

The selection of column dimension to be used in flash chromatography was done based on the sample size to be purified. In this work 30 cm × 1.5 cm or larger column was chosen. It was manually packed with silica gel 60 of an average particle size ranged between 40-63 μm, (60 g silica per 1 g of product). In the beginning, the sample was dissolved in a minimum amount of mobile phase. Then it was loaded onto the column. After that, the isocratic elution started using mixtures of methanol-dichloromethane with a ratio of 5:95, v/v (**1A** and **1B**), or toluene-ethyl acetate-methanol with a ratio of 8:6:1, v/v (**B**) as mobile phases. The flash chromatography was run at 10 cm min^-1^. The detection wavelength was 220 nm. The effluents from the column were collected into test tubes of 10 mL each. Fractions with same peak purity were combined, concentrated and then dried under reduced pressure. The collected extracts were determined by HPLC‏ (chromatograms are not shown).

## Results and Discussion

### Enzymatic hydrolysis

The enzymatic hydrolysis of alpha PL (1) utilizing two unique enzymes (Scheme 1) was investigated. Keeping in mind the end goal is to optimize the yield of the product where the deprotection took place at the position of C6. Moreover, the enzymatic hydrolysis of 2-acetamido-2-deoxy-1,3,4,6-tetra-O-acetyl α-D-glucopyranose (**1**), was carried out in a phosphate buffer solution, containing 10 or 20% acetonitrile. The later was done to guarantee full solubilization of the starting materials. The reactions took place at acidic pH to avoid any possibility for acyl group migration/movement from one -OH- to the next that could generate undesired *by-products*.^22^ Hydrolysis reactions were followed by TLC as well as HPLC.

For better screening of **A**, two different enzymes were used. The first one is called lipase obtained from CRGL immobilized on two different hydrophobic supports namely; DSEOD and OSCL. The second is ACEXE obtained from *Bacillus pumilus* which immobilized on acrylic resin and epoxy groups as functional groups.

The reaction continued with a high regioselectivity at carbon 6 position as indicated in Table 1. The results of the previous reaction was in agreement with the results reported for the hydrolysis of **A** that catalyzed by CRGL and immobilized at pH 4.^21,22^ CRGL immobilized on DSEOD showed a higher regioselectivity as well as activity in 24 h (98%) in comparison with the hydrolysis which catalyzed by CRGL immobilized on OSCL within 48h (27%) once the hydrolysis took place at pH 5. Actually, CRGL immobilized on these two hydrophobic matrixes revealed diverse region-selectivities and rate of biotransformation at the previous pH for **1A**.

In order to explore the reaction catalyzed by the biocatalyst CRGL which immobilized on DSEOD, an increasing concentration of **A**, to attain a preparative amount of **1A**, was used. Surprisingly, we noticed that the performance of CRGL was inversely proportional to substrate concentration in the range 64-98% yield. Precisely when the biocatalyst ACEXE was used, the hydrolysis of **A** proceeded with unexpected results (13% yield of **1A**, Table 1).

**Table 1:** Hydrolysis of substrate A catalyzed by different immobilized enzymes.

### HPLC method development 

Chromatographic methods are considered fundamental for monitoring the hydrolysis of drug substances or even synthesis of any new compound. This includes the analysis of intermediates and the synthesized reaction mixtures at particular intervals of time. It helps also in checking the purity, yield of reaction products generated and particular impurities which affect reaction. The current HPLC method has been adopted to follow/monitor the progress of reaction during the route of the hydrolysis of **A**, its conversion to **1A** and purity and yield of the **1A**.

A few chromatographic conditions have been investigated while developing the current HPLC method. For instance solvents, mobile phase, stationary phase, and detection wavelength. The chromatographic separation was accomplished using C18 column as it gave a base-line separation between the two substrates under examination (**A** and **1A**) and from *by-products* (chromatograms are not shown). The common challenge faced while screening the formation of **1A**, once the **A** subjected to hydrolysis, was to achieve complete base-line separation between the two substrates upon hydrolysis by ACEXE or CRGL. The cause of such challenge was attributed to similarity in structures as prescribed in Table 1 and from other *by-products* accordingly. After that, the reaction mixture was chromatographed on a reversed phase column and analyzed at 220 nm. Isocratic elution mode was applied which comprised of 15 and 20 % acetonitrile in phosphate buffer (10 mM, pH 4) as mobile phase for the hydrolysis of **1A** and **1B**, respectively.

After checking the reactions by RP-HPLC method, we noticed diverse *by-products* produced. These *by-products* were entitled by shorter retention times. This was attributed to the nature of the hydrophilic compounds (hydrolyzed monosaccharides in many positions). Specifically, the deprotection at C6 position. Indeed, after 24 h, the substrate was converted at 98% of the targeted monosaccharide **1A** and only 2% of *by-products* generated. As known, the absence of other peaks indicates the good purity of the isolated compounds. Then again, the hydrolysis of **A** catalyzed by ACEXE was very unspecific, producing only 13% of **1A** and 77% of other products (Table 1).

Next, the mild acyl migration/movement was investigated to get‏ the tetraacetylated glycopyranoses containing a free hydroxyl group at the C4 position. The last compound is considered useful being as a building block in the synthesis of PL 3. In this manner, the 6-hydroxy derivative **1A** (aqueous solution, pH 9 and 4°C) was converted to product **1B** and then isolated in a yield of 90% (scheme 1).

Starting from **A** using CRGL immobilized on DSEOD, the hydrolysis was performed at pH 5 and 25 °C. It helps in obtaining **1A** in a good yield. After that, separation of the immobilized enzyme by filtration was carried out. Next, the reaction conditions were altered by lowering the temperature to 4 °C and at the same time increasing pH to 9. Under these conditions used, a controlled acetyl group movement/migration from 4 to 6 position gave **1B** with 90% yield after isolation as indicated in Scheme 1. In order to quench the reaction, acidification at pH ranged between 4-5 was conducted. After that, extraction of 4-hydroxy **1B** in organic solvent was done. Then, flash chromatography was applied to purify the desired compound **1B**. The purified compound was isolated and characterized by RP-HPLC. Synthetic standards were used for identification purposes.

In addition, we described herein the optimization of a new method for the synthesis of PL. It represents a basic element in the structure of glycosidic antitumor carbohydrate. The 4-hydroxy derivative of the PL 2 (acceptor), once prepared using the chemoenzymatic process, was used as starting material in the glycosilation reaction for the synthesis of **B**. It was obtained through the reaction with 2,3,4 tetra-O-acetyl-α-D-galactopyranosyl trichloroacetimidate **2** prepared as in the protocol reported (donor).^23^

In glycosylation reaction, it is necessary for the reaction to take place that the donor molecule possesses in the anomeric position a good leaving group. Moreover, in the presence of promoting agent, it allows the formation of carbocationic intermediate that is able to react with the hydroxyl group of desired acceptor. The glycocidic bond must be in β configuration in order to get the desired **B**. Thus, it is deemed necessary to control bond configuration during the bond formation. This could be achieved through the neighboring group participation due to the presence of acetyl group at position 2 (**C**). This occurs through the formation of a cyclic structure called dioxolium ring which provides a steric shield for the face a of the molecule.‏ The importance of such formation of this intermediate permits the nucleophile (acceptor) to determine the nucleophilic attack from the b face of the electrophile (donor). Also, it allows the achievement of the chemical bond in the desired configuration.

To improve the yield of synthesis of **B,** it was analyzed under various reaction conditions. It was performed by coupling reaction between the two building blocks namely; **1B** and 2,3,4,6-tetra-O-acetyl-α-D-galactopyranosyl trichloroacetimidate **2** which prepared based on the protocol reported.^23^ Parameters such as the molar ratio (between donor 2 and acceptor **1B**), and temperature have been investigated. The results of the current study revealed that the yield of **B** was enhanced up to 95%. This is indicated in Table 2 and ascertained after the product of interest subjected to purification using flash chromatography utilizing the molar proportion of 2.5:1 (2:**1B**) and borontrifluoride diethyl etherate as promoting agent at room temperature (Table 2).

**Table 2:** Optimization of glycosylation reaction conditions.

### Flash chromatography method development (purification procedure)

As known, TLC is considered a straight approach for selecting of mobile phase to be used in silica gel flash chromatography.^14,24^ Furthermore, to start chromatographic purification, it is recommended to refer to protocols in literature as a guidance in selecting a versatile mobile phase and a column suitable to the solubility, molecular weight, and hydrophobic character of the analyte to be analyzed.^14,25,26^ In the current work, no reports have been published for flash purification of substrates **1B** and **B**. Therefore, development and determination of a suitable procedure is a challenging step of this work. Several mixtures of mobile phases were examined such as methanol/ ethyl acetate/toluene (1:6:8, v/v/v) and methanol/dichloromethane (5:95, v/v) to accomplish the purification of **1B** and **B**, respectively. The best organic solvent ratio to be used was determined by trial and error.

On the other hand, several of solvent systems were examined in TLC separation of the two substrates. For example, methanol/dichloromethane, ethyl acetate/chloroform, acetone/hexane, methanol/chloroform, methanol/ethyl acetate, acetone/chloroform, and methanol/toluene/ethyl acetate). The best separation achieved among the systems examined on TLC was accomplished as mentioned earlier.

### NMR spectroscopy

The final step is to verify the structure of **B** after purification using flash chromatography. Characterization has been done by ^1^HNMR spectra (spectra are not shown) while Figure 2 shows the mass spectrometry.

**Figure 2:** Mass spectrometry of the targeted compound (**B**).

^1^H-NMR (400 MHz, CDCl_3_): δ = 1.94-2.19 (8s, 24H, Ac), 3.85-3.92 (m, 3H, H-4, H-5 and H-5'), 4.06-4.16 (m, 3H, H-6a',H-6b' and H-6a), 4.38-4.44 (m, 2H, H-2, H-6b), 4.53 (d,1H, *J* = 8 Hz, H-1'), 4.98 (dd, 1H, H-3'), 5.15 (dd, 1H, H-2'), 5.25 (dd,1H, H-3), 5.39 (dd,1H, H-4'), 5.72 (d, 1H, *J* = 8.8 Hz, NH), 6.1 (d, 1H, *J* = 3.2, H-1).

MS (ESI)+ m/z: calcd for C_28_H_39_NO_18_: 677.21, found: 700.20 [M+Na]^+^

### 1D and 2D NMR study of B

The values of the ^1^H NMR chemical shifts for **B** in CDCl_3_ solution are reported in the previous section 3.4. Referring to the ^1^H NMR chemical shifts for **B** illustrated eight signals appeared as singlet in the most high-field region of δ = 1.94 ppm, δ = 1.98 ppm, δ = 2.06 ppm, δ = 2.08 , δ = 2.11, δ = 2.13, δ = 2.16, δ = 2.19, for 8s, 24H, and COCH_3_, respectively. This is due to the protons in CH_3_ presents in COCH_3_ groups (8s, 24H, COCH_3_). Additionally, a multiplet which appeared in the high-field region at δ = 3.85-3.92 ppm‏ was assigned to the three protons namely; m, 3H, H-4, H-5‏ and H-5'. A resonating, which appeared as multiplet at the range of δ = 4.06‏ -‏ 416 ppm were assigned‏ for protons (m, 3H, H-6a', H-6b' and H-6a). On the other hand, the multiplet at the range of δ = 4.38 - 4.44 ppm was assigned to the protons namely; m, 2H, H-2, H-6b. Moreover, proton H-1'was assigned for the doublet which appeared at the range of δ = 4.53 ppm (d, 1H, *J* = 8 Hz, H-1'). The doublet of doublet at δ = 4.98 dd ppm, was assigned to the proton (dd, 1H, H-3'). Also, the ^1^H NMR data showed that the signals of the protons due to 1H, H-2' was assigned as doublet of doublet at δ = 5.15 ppm (dd, 1H, H-2'). The signal of proton due to 1H, H-3 appeared at δ = 5.25 ppm (dd, 1H, H-3). The signal of proton due to 1H, H-4' appeared at δ = 5.39 ppm (dd, 1H, H-4'). Additionally, the signal of proton due to 1H, NH appeared at δ = 5.72 ppm (d, 1H, *J* = 8.8 Hz, NH) and the signal of H-1 appeared as a doublet at δ = 6.1 ppm (d, *J* = 3.2 Hz, 1H, H-1).

## Conclusion

An efficient chemoenzymatic procedure in order to optimize the preparation of PL 3 containing acetyl ester as extraordinary protecting group is presented herein. Compound **B** is a significant intermediate for the synthesis of pharmacologically active compound (e.g., complex oligosaccharides for biochemical, biophysical, or biological examinations and so on).^27^ Immobilized lipase from CRGL has been contrasted and the immobilized ACEXE from *Bacillus pumilus*, with regard to their exploitation in biotransformation of PL 1. CRGL was immobilized on two diverse solid supports, to be specific; OSCL, and DSEOD including hydrophobic adsorption. While ACEXE was covalently linked to the matrix by means of oxirane-groups sepabeads. The hydrolysis of **A** which catalyzed by CRGL affirmed that the performance of the immobilized enzyme is strongly affected by the kind of support. Lipase immobilized on DSEOD was more active and regioselective than the lipase immobilized on OSCL, producing **1A** in 98% at 100% of conversion, and 27% at 75% of conversion of **A**, respectively.

Besides, reaction monitoring utilizing HPLC proposes more exact information than spectroscopic methods. For instance, it gives the content of starting material, product and the impurities during the course of the reaction. Besides, these outcomes help researchers and scientist to optimize and enhance the reaction conditions, improve the quality and quantity of the product. Moreover, we conclude that HPLC is considered as an effective and important tool for *in-process* analysis. It aids to increase the quality, quantity of the products and reduce the manufacturing cost. In this work, an isocratic HPLC method for controlling the hydrolysis of **A** to **1A** with the guide of ACEXE and CRGL-OSCL was developed. The newly developed method was observed to be simple, and able of separating the two substrates in addition to all *by-products* connected with the process of hydrolysis. In this way, this method can be valuable for *in-process* control and additionally quality affirmation in the pharmaceutical industry.

## Acknowledgments

This work was funded by Drug Sciences Department, Pavia University, Italy.

## Ethical Issues

Not applicable.

## Conflict of Interest

The authors declare no conflict of interests.
